The article "Fibulin-4 is associated with prognosis of endometrial cancer patients and inhibits cancer cell invasion and metastasis via Wnt/β-catenin signaling pathway" was retracted in 2026. Reasons: plagiarism; duplicated images; overlap with other authors' work.

# Fibulin-4 is associated with prognosis of endometrial cancer patients and inhibits cancer cell invasion and metastasis via Wnt/β-catenin signaling pathway

**DOI:** 10.18632/oncotarget.15086

**Published:** 2017-02-04

**Authors:** Tiantian Wang, Mei Wang, Shuang Fang, Qiang Wang, Rui Fang, Jie Chen

**Affiliations:** ^1^ Department of Maternal and Child Health, School of Public Health, Shandong University, Jinan 250012, China; ^2^ Pharmacy Department, Shandong Provincial Hospital affiliated to Shandong University, Jinan 250012, China; ^3^ Biochemistry and Molecular Biology, Georgetown University, Georgetown, Washington D.C 20057, USA; ^4^ Department of Obstetrics and Gynecology, The Second Hospital affiliated to Jilin University, Jilin 130000, China; ^5^ Clinical Medicine, School of Medicine, Shandong University, Jinan 250012, China

**Keywords:** fibulin-4, endometrial cancer, invasion, metastasis, epithelial-mesenchymal transition (EMT)

## Abstract

Fibulin-4, an extracellular glycoprotein, which plays significant roles in elastic fiber assembly, is correlated to the progression of some cancers. However, the role of fibulin-4 in endometrial cancer cell invasion and metastasis remains unexplored. In our study, fibulin-4 expression was assessed by immunohistochemistry (IHC) and reverse transcription-quantitative polymerase chain reaction (RT-qPCR) in normal endometrial tissues and endometrial carcinoma tissues. Using single cell cloning, strongly, and weakly, invasive subclones were derived from KLE and Ishikawa endometrial carcinoma cell lines. RT-qPCR, western blotting, and immunocytochemistry (ICC) were used to assess mRNA and protein expressions of fibulin-4 in primary cultured endometrial cells, 4 types of endometrial cancer cell lines, and the different invasive subclones. Using lentivirus transfection, fibulin-4 shRNA and pLVX-fibulin-4 were constructed and used to infect the strongly and weakly invasive subclones. The effects of fibulin-4 on the biological characteristics of endometrial carcinoma cells were detected by cell functional assays *in vitro* and *in vivo*. Using Wnt signaling pathway inhibitor XAV-939 and activator LiCl, we detected the role of fibulin-4 in the Wnt/β-catenin pathway and the relationship with epithelial to mesenchymal transition (EMT). Fibulin-4 was decreased in endometrial carcinoma tissues, and loss of fibulin-4 expression was significantly related with poor differentiation, lymph node metastasis, and poor prognosis of endometrial carcinoma. Fibulin-4 significantly inhibited endometrial carcinoma cell proliferation, invasion, metastasis, and EMT through the Wnt/β-catenin pathway. Fibulin-4 has the ability to suppress endometrial cancer progression. These results can contribute to the development of a new potential therapeutic target for patients with endometrial carcinoma.

## INTRODUCTION

Endometrial carcinoma is the second most common malignant tumor occurring in the female genital tract [1]. Although early-stage endometrial cancer generally has a favorable outcome, up to 30% of endometrial cancer patients are diagnosed with International Federation of Gynecology and Obstetrics (FIGO) stage III or IV, and have a relatively poor prognosis, with local or extra-pelvic metastasis, and even distant metastasis [2, 3]. Metastasis causes most cancer deaths [4], so there is an urgent requirement for exploring the mechanism of tumor invasion and metastasis to further elucidate the progression of cancers. Recently, many biomarkers that are related with the development of endometrial carcinoma have been evaluated; however, no information has been found regarding the function of fibulin-4 in endometrial cancer cell invasion and metastasis.

Fibulins, encoded by the FBLN genes, are extracellular matrix proteins sustaining the integrity and stability of basement membranes, elastic fibers [5], and loose connective tissue [6]. Presently, the fibulin family contains seven members: fibulin-1, fibulin-2, fibulin-3, fibulin-4, fibulin-5, fibulin-6, and fibulin-7 [7]. Fibulin family members have been observed to participate in modulating cell morphology, growth, adhesion, and motility, which is intimately related to the occurrence and development of various kinds of cancers [8]. Fibulin-4, also called endothelial growth factor (EGF)-containing fibulin-like extracellular matrix protein 2 (EFEMP2), and mutant p53 binding protein 1 (MBP1) [9], are critical molecules for elastic fiber assembly [5]. Meanwhile, fibulin-4 is associated with many diseases, including cutis laxa [10], aortic dissection [11], osteoarthritis [12], and cancer [8]. At present, research on the correlation between fibulin-4 and tumors is still in the initial stage. The role of fibulin-4 in endometrial cancer cell growth and metastasis remains unexplored. This is the first study to clarify the effects of fibulin-4 on the progression of endometrial cancer and the function of fibulin-4 in endometrial cancer cell proliferation, invasion, and metastasis.

## RESULTS

### Fibulin-4 expression in human endometrial tissues

As shown in Figure 1, high fibulin-4 protein expression was detected in normal endometrial tissue, especially in the stroma and the endometrial cell cytoplasm (Figure 1A, 1B). However, in most endometrial carcinomas, fibulin-4 immunoreactivity was very low. We found that the expression of fibulin-4 in the cancer stroma was reduced or even disappeared with the increase of malignant degree of endometrial carcinoma. Compared to the well differentiated tumor group (Figure 1E), low expressions of fibulin-4 were found in the poor differentiated tumor group (Figure 1F), mainly in the cell cytoplasm, not stroma. Moreover, low fibulin-4 protein expression was positively correlated with advanced stage, and lymph node metastasis, of endometrial carcinomas (Table 1). Similar results were observed with RT-qPCR. Significantly, high fibulin-4 mRNA expression was seen in normal endometrial tissues; however, there was a very low level of fibulin-4 mRNA expression in endometrial carcinomas. Moreover, the low mRNA expression of fibulin-4 was also positively correlated with poor tumor differentiation, advanced stage, and lymph node metastasis of endometrial carcinomas (Table 2). Overall survival (OS) was defined as the interval between the date of diagnosis and the date of death from any cause or last patient visit. Progression-free survival (PFS) was defined as the time from diagnosis to any type of tumor relapse either local or distant. OS and PFS analyses were estimated using the Kaplan-Meier statistical method to assess the prognostic value of fibulin-4 in endometrial carcinomas. The result showed that patients with high fibulin-4 expression had a much better prognosis than those with low fibulin-4 expression (Figure 1K, 1L).

**Figure 1:** Expressions of fibulin-4 in human endometrial tissues The proliferative stage of normal human endometrium (**A**), the secretory phase of normal human endometrium (**B**), human endometrium with complex hyperplasia (**C**), particular atypical endometrial hyperplasia (**D**), well differentiation of endometrial carcinoma (**E**), poor differentiation of endometrial carcinoma (**F**), the area of squamous differentiation (**G**), the clear cell carcinoma (**H**) and the serous carcinoma (**I**) were measured by IHC. (Magnification×200). (**J**) Western blot analysis was performed to detect fibulin-4 in a set to paired normal-tumor tissue samples. (**K**) Kaplan-Meier curve showing overall survival. (**L**) Kaplan-Meier curve showing progression-free survival. Patients with low fibulin-4 expression (green line, *n* = 171) had much worse prognosis than those with high fibulin-4 expression (blue line, *n* = 29).

**Table 1:** Protein expression of fibulin-4 in human endometrial tissues

	*N*	Fibulin-4 low (−/+)		Fibulin-4 high (++/+++)		χ^2^	*P*-value
		*n*	(%)	*n*	(%)		
Normal	40	2	5	38	95	103.3	*P* < 0.05
Carcinoma	200	171	85.5	29	14.5		
Pathological type						12.7	*P* > 0.05
*Endometrioid*	165	143	86.7	22	13.3		
*Serous*	20	16	80	4	20		
*Clear-cell*	15	12	80	3	20		
Cell differentiation						14.5	*P* < 0.05
*Well*	96	75	78.1	21	21.9		
*Poor*	69	68	98.6	1	1.4		
Tumor stage						34.1	*P* < 0.05
*Stage I*	78	58	74.4	20	25.6		
*Stage II*	65	57	87.6	8	12.3		
*Stages III and IV*	57	56	98.2	1	1.8		
Nodal status						20.0	*P* < 0.05
*Positive*	78	74	94.9	4	5.1		
*Negative*	122	97	79.5	25	20.5		

**Table 2:** mRNA expression of fibulin-4 in human endometrial tissuesxs

	*N*	fibulin-4 mRNA Ratio of fibulin-4/β-actin	*P*
Normal	40	0.0985 ± 0.0083	
Carcinoma	200	0.0303 ± 0.0026	< 0.05
Pathology type			> 0.05
*Endometrioid*	165	0.0478 ± 0.0034	
*Serous*	20	0.0391 ± 0.0036	
*Clear-cell* Cell differentiation	15	0.0256 ± 0.0028	< 0.05
*Well*	116	0.0257 ± 0.0078	
*Poor*	84	0.0068 ± 0.0013	
Tumor stage			< 0.05
*Stage I*	78	0.0448 ± 0.0057	
*Stage II*	65	0.0259 ± 0.0041	
*Stages III and IV*	57	0.0086 ± 0.0014	
Nodal status			< 0.05
*Positive*	78	0.0058 ± 0.0016	
*Negativ*e	122	0.0379 ± 0.0035	

### Acquisition of endometrial epithelial cells and stromal cells

As shown in Supplementary Figure 1, under the inverted microscope, the endometrial epithelial cells were observed to grow into a spiral-packed, monolayer cell colony that was closely arranged. Using ICC, cytokeratin (sc-57004, Santa Cruz) staining was positive in the cytoplasm of epithelial cells. However, endometrial stromal cells were mostly spindle-shaped and vimentin (sc-373717, Santa Cruz) staining was positive in the cytoplasm of stromal cells. With continuing cell passage, endometrial epithelial cells died, while endometrial stromal cells could be passaged for approximately 5 generations.

### Establishment of strongly invasive subclones and weakly invasive subclones

As shown in Supplementary Figure 2, using the single cell cloning technique, a total of 28 KLE subclones and 23 Ishikawa subclones were obtained. KLE-1 and ISK-1, which had the highest migration rates (19.75 ± 0.52 μm/s and 18.82 ± 0.46 μm/s) showed higher proliferation and invasive abilities than KLE-28 and ISK-23, which had the lowest migration rates (8.77 ± 0.16 μm/s and 7.58 ± 0.13 μm/s). The *in vitro* growth abilities of KLE-1 and ISK-1 were higher than those of KLE-28 and ISK-23. In the cell migration and Matrigel invasion assays, the average migration and invading cell numbers of KLE-1 and ISK-1 were much higher than those of KLE-28 and ISK-23. In tumor xenograft experiments, KLE-1 and ISK-1 cells were injected subcutaneously in nude mice to form 100% tumors, which grew rapidly. However, the tumor forming rates of KLE-28 and ISK-23 were only about 50%, and the tumors grew very slowly. The volumes of tumors formed by KLE-1 and ISK-1 were 540.71 ± 37.54 mm^3^ and 510.52 ± 34.31 mm^3^, respectively, much higher than those formed by KLE-28 and ISK-23 (49.23 ± 3.65 mm^3^ and 35.91 ± 4.73 mm^3^, respectively, *P* < 0.01).

### Different proliferation and invasion abilities of 4 types of human endometrial cancer cell line

Compared to Ishikawa and HEC-1B cells, KLE and HEC-1A cells had higher proliferation abilities (Figure 2A). In the soft agar colony formation assay (Figure 2B, 2C); the colony numbers formed by KLE and HEC-1A cells (45.04 ± 4.62 and 40.32 ± 3.49) were significantly higher than those formed by Ishikawa and HEC-1B cells (8.16 ± 1.33 and 8.76 ± 2.27, *P* < 0.01). Accordingly, in the cell migration assay and the Matrigel invasion assay (Figure 2D, 2E), KLE and HEC-1A cells were also detected to have stronger migration and invasion abilities. In the cell migration assay (Figure 2F), the average migrating cell counts of KLE and HEC-1A cells were much higher than those of Ishikawa and HEC-1B cells (387.27 ± 32.72 and 354.33 ± 27.47 vs. 132.13 ± 18.61 and 128.07 ± 19.43, *P* < 0.05). Similar results were also detected in the Matrigel invasion assay (Figure 2G); the average invading cell counts of KLE and HEC-1A cells were much higher than those of Ishikawa and HEC-1B cells (168.25 ± 12.29 and 148.07 ± 15.74 vs. 44.34 ± 6.83 and 52.18 ± 7.21, *P* < 0.05). In conclusion, KLE and HEC-1A cells had stronger proliferation and invasion abilities, in contrast with Ishikawa and HEC-1B cells.

**Figure 2:** Different proliferation, migration and invasion abilities of 4 types of human endometrial cancer cell lines (**A**) The growth curves of human endometrial cancer cells showed that KLE and HEC-1A cells had higher proliferation abilities compared to Ishikawa and HEC-1B cells. (**B**) The colony numbers formed by KLE and HEC-1A cells were significantly higher than those formed by Ishikawa and HEC-1B cells. (**C**) The colony images of human endometrial cancer cells as examined by soft agar colony formation assay. (**D**) The images of cells migrating PVPF filters as examined by cell migration assay using Boyden chambers. (**E**) The images of cells invading Matrigel-coated membranes as examined by cell invasion assay using Boyden chambers. (**F**) The average migrating cell counts of KLE and HEC-1A cells were much higher than those of Ishikawa and HEC-1B cells. (**G**) The average invading cell counts of KLE and HEC-1A cells were much higher than those of Ishikawa and HEC-1B cells. (Magnification ×200).*P < 0.05 versus control.

### Fibulin-4 expression in human endometrial cell lines, strongly invasive subclones, and weakly invasive subclones

As shown in Figure 3, the strongest expression of fibulin-4 was detected in normal endometrial cells. And compared to Ishikawa and HEC-1B cells, fibulin-4 was weakly expressed in KLE and HEC-1A cells, which had higher proliferation and invasion abilities. In contrast with the weakly invasive subclones (Figure 4), low fibulin-4 expression was also found in strongly invasive subclones KLE-1 and ISK-1. These results were consistent with those obtained from endometrial tissues, which indicated that low expression of fibulin-4 was closely related to the invasion of endometrial carcinoma.

**Figure 3:** Fibulin-4 expressions in endometrial carcinoma cells and normal endometrial cell Fibulin-4 expressions of KLE, Ishikawa, HEC-1A, HEC-1B and normal endometrial cells as measured by (**A**) ICC staining (Magnification×200), (**B**) western blot and (**C**) q-RT-PCR. The strongest expression of fibulin-4 was detected in normal endometrial cells, and compared to Ishikawa and HEC-1B cells, fibulin-4 was weakly expressed in KLE and HEC-1A cells, which had higher proliferation and invasion abilities. *P < 0.05 versus control.

**Figure 4:** Fibulin-4 expressions in strongly invasive subclones and weakly invasive subclones Fibulin-4 expressions in strongly invasive subclones and weakly invasive subclones as measured by (**A**) ICC staining (Magnification×200), (**B**) q-RT-PCR and (**C**) western blot. In contrast with the weakly invasive subclones, low fibulin-4 expression was found in strongly invasive subclones KLE-1 and ISK-1.*P < 0.05 versus control.

### Decreased and increased expression of fibulin-4 in weakly invasive subclones and strongly invasive subclones

In order to further investigate the possible function of fibulin-4 in endometrial cancer cell proliferation and invasion, using RNA interference, fibulin-4 expression was decreased in the weakly invasive subclones KLE-28 and ISK-23. Meanwhile, using lentivirus transfection, fibulin-4 expression was increased in the strongly invasive subclones KLE-1 and ISK-1. After viral infection, the changes in fibulin-4 expression were confirmed by real-time q-RT-PCR, western blot and ICC at both mRNA and protein levels, which indicated high efficiency in the transfection experiments (Figure 5).

**Figure 5:** Identification of the transfection efficiencies after lentivirus-mediated transfection Fibulin-4 expressions in lentivirus-infected cells as measured by (**A**) western blot, (**B**) ICC staining (Magnification ×200), and (**C**) q-RT-PCR. After viral infection, fibulin-4 expression was decreased in the weakly invasive subclones KLE-28 and ISK-23, meanwhile, fibulin-4 expression was increased in the strongly invasive subclones KLE-1 and ISK-1.*P < 0.05 versus control.

### Effects of fibulin-4 on endometrial cancer cell proliferation

The cell proliferation abilities of weakly invasive subclones KLE-28 and ISK-23 were significantly promoted by fibulin-4 knockdown; accordingly increased fibulin-4 could inhibit the proliferation ability of strongly invasive subclones KLE-1 and ISK-1 (Figure 6A). In the soft agar colony formation assay, colony forming efficiencies of fibulin-4 shRNA-infected cells were increased, and correspondingly, increased fibulin-4 could decrease the colony forming efficiency of the strongly invasive subclones KLE-1 and ISK-1 (Figure 6B). There were no significant differences between non-infected groups and negative control groups.

**Figure 6:** Effects of fibulin-4 on cell proliferation and colony formation abilities (**A**) Knockdown of fibulin-4 promoted cell proliferation abilities of the weakly invasive subclones, meanwhile, over-expression of fibulin-4 inhibited cell proliferation abilities of the strongly invasive subclones. (**B**) Fibulin-4 knockdown increased the colony forming capacities of weakly invasive subclone, while over-expression of fibulin-4 decreased the colony forming capacities of strongly invasive subclone. *P < 0.05 versus control.

### Effects of fibulin-4 on endometrial cancer cell migration and invasion

As shown in Figures 7 and 8, knockdown of fibulin-4 increased the invasion and migration abilities of the weakly invasive subclones KLE-28 and ISK-23, and the invasion and migration ability of strongly invasive subclones KLE-1 and ISK-1 were significantly inhibited by fibulin-4 upregulation. There was no significant difference between negative controls and non-infected groups.

**Figure 7:** Effects of fibulin-4 on cell migration abilities (**A**) Cell migration images of lentivirus-infected cells as measured by Boyden chambers without Matrigel. (Magnification ×200). (**B**) Fibulin-4 knockdown promoted cell migrating abilities, while fibulin-4 over-expression suppressed cell migrating abilities. *P < 0.05 versus control.

**Figure 8:** Effects of fibulin-4 on cell invasion abilities (**A**) Cell invasion images of lentivirus-infected cells by Boyden chambers coated with Matrigel. (Magnification ×200). (**B**) Fibulin-4 knockdown promoted cell invading abilities, while fibulin-4 over-expression suppressed cell invading abilities. *P < 0.05 versus control.

### Effects of fibulin-4 on tumor growth in xenograft model

Fibulin-4 shRNA-infected KLE-28 cells and negative control KLE-28 cells, as well as pLVX-fibulin-4-infected KLE-1 cells and negative control KLE-1 cells, were inoculated subcutaneously or through the tail veins into 5 nude mice each. The tumor formation rates of fibulin-4 shRNA-infected KLE-28 cells and negative control KLE-1 cells were 100%, with relatively fast tumor growth. While only 40% tumor formation rates were observed in pLVX-fibulin-4-infected KLE-1 cells and negative control KLE-28 cells. Moreover, the average tumor volumes of fibulin-4 shRNA infected KLE-28 cells and negative control KLE-1 cells were much higher than those formed by negative control KLE-28 cells and pLVX-fibulin-4-infected KLE-1 cells (513.94 ± 30.54 mm^3^ vs. 99.43 ± 9.02 mm^3^ and 546.78 ± 32.64 mm^3^ vs. 104.25 ± 8.13 mm^3^, *P* < 0.01) (Figure 9A, 9B). Collectively, fibulin-4 could inhibit tumor formation and growth *in vivo*. The pLVX-fibulin-4-infected group and the weakly invasive subclone group had no lung metastasis; however, the lung metastasis rates of the fibulin-4 knockdown group and the strongly invasive group were 80% and 100%, respectively (Figure 9C). In conclusion, fibulin-4 can be a promising inhibitor of endometrial cancer progression.

**Figure 9:** Effects of fibulin-4 on tumor growth and lung metastasis in nude mice (**A**) Tumor growths of lentivirus-infected cells were observed continuously for 8 weeks. The average tumor volumes of fibulin-4 shRNA infected KLE-28 cells and negative control KLE-1 cells were much higher than those formed by negative control KLE-28 cells and pLVX-fibulin-4-infected KLE-1 cells. (**B**) Photograph of xenografts dissected from nude mice after subcutaneous inoculation. (**C**) H&E staining were performed on lung metastasis after inoculation through tail vein. The pLVX-fibulin-4-infected group and the weakly invasive subclone group had no lung metastasis; however, the lung metastasis rates of the fibulin-4 knockdown group and the strongly invasive group were 80% and 100%, respectively. (Magnification ×200). *P < 0.05 versus control.

### Effects of fibulin-4 on EMT genes and normal endometrial fibroblasts

It is well known that EMT is correlated with cancer invasion and metastasis. So we suspected that fibulin-4 could produce an effect on the EMT genes. The effects of fibulin-4 knockdown and upregulation on several key EMT genes, including E-cadherin, N-cadherin, vimentin, snail, slug and twist, were investigated using real-time q-RT-PCR and western blot. The results showed that fibulin-4 knockdown significantly decreased the expression of E-cadherin, and increased the expression of N-cadherin, vimentin, snail, slug and twist (Figure 10); meanwhile fibulin-4 up-regulation could increase the expression of E-cadherin, and decrease the expression of N-cadherin, vimentin, snail, slug and twist (Figure 11). In conclusion, fibulin-4 could inhibit the invasion and metastasis of endometrial cancer cells by preventing the expression levels of EMT genes. In order to examine the effect of fibulin-4 on normal endometrial fibroblasts, we co-cultured normal endometrial fibroblasts and pLVX-fibulin-4-infected KLE-1 for 24h, 48h, and72h. The results showed that the fibroblasts markers vimentin and alpha-smooth muscle actin were significantly decreased with the extension of co-culture time. These results indicated that fibulin-4 as an extracellular matrix protein, could play an important role in endometrial fibroblasts (Figure 11).

**Figure 10:** Effects of fibulin-4 knockdown on EMT genes correlated to tumor progression After RNA interference, EMT markers, including E-cadherin, N-cadherin, vimentin, Snail Slug and Twist as measured by (**A**) Western blot and (**B**) real-time qPCR in the fibulin-4 shRNA infected groups. The results showed that fibulin-4 knockdown significantly decreased the expression of E-cadherin, and increased the expression of N-cadherin, vimentin, snail, slug and twist. *P < 0.05 versus control.

**Figure 11:** Effects of fibulin-4 over-expression on EMT genes correlated to tumor progression After transfection, EMT markers, including E-cadherin, N-cadherin, vimentin, Snail Slug and Twist as measured by (**A**) Western blot and (**B**) real-time qPCR in the pLVX-fibulin-4 infected groups. The results showed that fibulin-4 up-regulation could increase the expression of E-cadherin, and decrease the expression of N-cadherin, vimentin, snail, slug and twist. (**C**) After co-culturing normal endometrial fibroblasts and pLVX-fibulin-4-infected KLE-1 for 24 h, 48 h, and72 h, the fibroblasts markers vimentin and alpha-smooth muscle actin (α-SMA) were significantly decreased with the extension of co-culture time. *P < 0.05 versus control.

### Effects of fibulin-4 on the Wnt/ β-catenin pathway

A variety of pathways, including the Wnt/β-catenin and Notch pathways, induce EMT and reduce the expression of E-cadherin. So we utilized several key genes of the Wnt/β-catenin pathway, including β-catenin, C-myc, and cyclin D1, and the Notch pathway, including NICD, HES 1, and HEY L in the lentivirus transfection system (Figure 12). The results showed that there were no obvious effects on the Notch pathway, when fibulin-4 was up- or down- regulated. However, in the Wnt/β-catenin pathway, fibulin-4 knockdown increased the expression of β-catenin, C-myc, and cyclin D1, activating the Wnt/β-catenin pathway, and at the same time, reduced the expression of E-cadherin, and promoted EMT. Meanwhile, fibulin-4 upregulation decreased the expression of β-catenin, C-myc, and cyclin D1, deactivated the Wnt/β-catenin pathway, increased the expression of E-cadherin, and inhibited EMT. Using Wnt signaling pathway inhibitor XAV-939 (5, 10, and 20 μmol/L) and activator LiCl (5, 10, and 20 μmol/L) we treated the fibulin-4 shRNA-infected cells and pLVX-fibulin-4-infected cells, for 48 h. We found that Wnt signaling pathway inhibitor XAV-939 could significantly inhibit the Wnt/β-catenin pathway, and EMT, both of which were activated by fibulin-4 knockdown; at the same time, Wnt signaling pathway activator LiCl could promote the Wnt/β-catenin pathway and EMT, which were deactivated by fibulin-4 upregulation. We observed concentration-dependent increases with the increase in the dose. These results indicated that fibulin-4 could inhibit endometrial cancer cell migration and invasion by preventing EMT via the Wnt/β-catenin pathway (Figure 13).

**Figure 12:** Effects of fibulin-4 on the Wnt/β-catenin and Notch pathways (**A**) Fibulin-4 knockdown increased the expression of β-catenin, C-myc, and cyclin D1, activating the Wnt/β-catenin pathway, but had no obvious effects on the Notch pathway. (**B**) Fibulin-4 upregulation decreased the expression of β-catenin, C-myc, and cyclin D1, deactivated the Wnt/β-catenin pathway, but had no obvious effects on the Notch pathway.

**Figure 13:** Inhibition and promotion the Wnt/β-catenin pathway (**A**) In the fibulin-4 shRNA-infected cells, Wnt signaling pathway inhibitor XAV-939 could significantly inhibit the Wnt/β-catenin pathway and EMT, both of which were activated by fibulin-4 knockdown. (**B**) In the pLVX-fibulin-4-infected cells, Wnt signaling pathway activator LiCl could promote the Wnt/β-catenin pathway and EMT, both of which were deactivated by fibulin-4 upregulation.

## DISCUSSION

In our study, we initially detected that low expression of fibulin-4 was associated with poor clinical pathological characteristics of endometrial cancer, and fibulin-4 could inhibit endometrial cancer cell proliferation, invasion and metastasis by preventing EMT via the Wnt/β-catenin pathway.

By RT-qPCR, western blot, and IHC or ICC, we found that the expression of fibulin-4 in normal endometrial tissues and cells was much higher than that in endometrial cancer tissues and cells. Compared to strongly invasive endometrial cancer cell lines and subclones, fibulin-4 was detected as highly expressed in the low metastatic cell lines and subclones. Moreover, high expression of fibulin-4 was found in the endometrial cancer specimen tissues with well differentiation and negative lymph node status. Until now, in prostate cancer [5], fibulin-4 was found weakly expressed in carcinoma cell lines compared to normal prostate epithelial cells, similar to our findings for endometrial cancer. On the other hand, in osteosarcoma [13], the expression of fibulin-4 was high in the osteosarcoma clinical specimens and cell lines, but not in normal specimens and cell lines. In gliomas, the expression of fibulin-4 was significantly increased in glioma tissues compared to non-tumorous brain tissues [14]. In the studies of other gynecologic tumors, such as cervical carcinoma and ovarian cancer, overexpressed fibulin-4 was also found in cancer tissues and strongly invasive cells, and high expression of fibulin-4 was associated with tumor progression and poor prognosis [9, 15]. The dysregulation of certain fibulins occurred in a range of human cancers. Indeed, both tumor suppressive and oncogenic activities had been reported for members of the fibulin family. Fibulin-1 was overexpressed in epithelial ovarian and breast cancers. In estrogen receptor (ER)-positive ovarian and breast cancer cell lines, fibulin-1 mRNA levels are markedly increased by estrogens [16]. However, in gastric cancer [17], lung adenocarcinoma [18], colorectal cancer [19], bladder cancer [20], renal cell carcinoma [21], and hepatocellular carcinoma [22], fibulin-1 acted as a tumor suppressor and was significantly down-regulated in carcinoma, low fibulin-1 protein expression was associated with poor tumor differentiation and advanced N stage. Fibulin-2 was a driver of malignant progression in lung adenocarcinoma and played an unexpected role in collagen cross-linking and tumor cell adherence to collagen [23]. But in nasopharyngeal carcinoma [24] and breast cancer [25], fibulin-2 as a tumor suppressor gene, could inhibit cell proliferation, migration, invasion and angiogenesis *in vitro*. Fibulin-3 was reported to be highly expressed in ovarian cancer [26], osteosarcoma [27], pancreatic cancer [28], cervical cancer [29], and glioma [30], and promoted tumor development. However, in hepatocellular carcinoma [31], gastric cancer [32], lung cancer [33], endometrial carcinoma [34], breast cancer [35], nasopharyngeal carcinoma [36], and glioblastoma [37], fibulin-3 was downregulated, and could inhibit tumor cell proliferation, invasion, and metastasis. Fibulin-5 was widely considered a tumor suppressor gene that inhibited tumor growth, invasion, and angiogenesis in the development of most tumors [38–42]. Distinct fibulins are subjected to multiple expression regulations with either anti or pro-tumor effects, and the role of fibulins in tumor progression may display tissue specificity [8].

Until now, the mechanism of fibulin-4 in endometrial cancer cell proliferation, invasion, and metastasis remains unclear. It is well known that EMT correlates to the progression of many epithelial cancers, which is closely associated to the dissemination and invasion of malignant epithelial cells [43–45]. So we wondered whether it is possible for fibulin-4 to prevent the invasion and metastasis of endometrial cancer cells by inhibiting EMT. Our related results confirmed our suspicions. Knockdown of fibulin-4 suppressed epithelial marker E-cadherin expression, and increased the expression of interstitial markers N-cadherin and vimentin; meanwhile upregulated fibulin-4 resulted in increased E-cadherin expression, and decreased N-cadherin and vimentin expression. The transcription factors, including Snail (Snail-1), Slug (Snail-2), and Twist, which could inhibit the expression of E-cadherin and induce EMT, were all found to be increased when fibulin-4 was knocked down, and decreased when fibulin-4 was upregulated. All these data simultaneously indicated that fibulin-4 could inhibit EMT, and thereby prevent the invasion and metastasis of endometrial cancer cells. The relationship between fibulin-4 and EMT has not yet been reported in other tumors.

The Wnt/β-catenin signaling pathway plays an important role in cell proliferation, differentiation, and apoptosis, and is important for the occurrence, invasion, and metastasis of tumors. Disturbance of the Wnt signal pathway is related to a high incidence of many kinds of human cancers [46–49]. In our study, we found that fibulin-4 knockdown could activate the Wnt signaling pathway and promote EMT; on the other hand, increased fibulin-4 could inhibit the Wnt signaling pathway and prevent EMT. Furthermore, these processes could be reversed by the Wnt signal pathway activators or inhibitors. However, this phenomenon was not observed in the Notch signaling pathway when the lentivirus transfections of the fibulin-4 gene were conducted. Hence, we believed that fibulin-4 could inhibit EMT through the Wnt/β-catenin signaling pathway. In human osteosarcoma [13], the researchers obtained similar results, in that fibulin-4 showed no obvious effect on Notch signaling, but activated Wnt/β-catenin signaling. The difference was that fibulin-4 acted as an oncogene in osteosarcoma, and treatment with fibulin-4 protein significantly enhanced the activity of the Wnt/β-catenin pathway. In conclusion, in endometrial cancer, fibulin-4 acts as a tumor suppressor, and inhibits cancer cell invasion and metastasis by preventing EMT proceeding through the Wnt/ β-catenin pathway.

Fibulin-3 and fibulin-4 share high homology with > 50% amino acid identity in structure, and each has a modified cbEGF domain, with an insertion of 28 to 88 amino acids [50]. In the study on cervical carcinoma [9, 51] and ovarian cancer [15, 52], fibulin-4 and fibulin-3 were both found to be highly increased in cancer tissues and cells, and this was closely related to the malignant phenotype of the tumor. However, in endometrial carcinoma, fibulin-3 was decreased, inhibited tumor cell proliferation and invasion, and prevented epithelial-mesenchymal transition via Wnt/β-catenin signaling [53, 54]. We observed similar results with Fibuin-4 as well. The role of fibulin-4 in different gynecological tumors is different, perhaps because the tumor microenvironment influences the function of tumorigenic genes [55]. Fibulin-3 and fibulin-4 are very similar in structure and function; hence, we speculate that they may be functionally coordinated; however, this hypothesis requires further experimental evidence.

In conclusion, the expression of fibulin-4 was negatively correlated with the malignant phenotype of endometrial cancer cells. Fibulin-4 may have the ability to suppress endometrial cancer cell invasion and proliferation. We believe that this study on fibulin-4 may contribute to the more effective treatment for inhibiting invasion and metastasis of endometrial cancer.

## MATERIALS AND METHODS

### Human primary endometrial cell isolation and culture

Primary normal endometrial cells were obtained from surgically resected endometrial hysterectomy specimens using the trypsin method, which utilizes the enzymatic activity of trypsin to facilitate the separation of cells and primary cell outgrowth. Human endometrial tissue was placed in DMEM/F12 (Gibco BRL, Rockville, MD) supplemented with 1% antibiotics (HyClone, Logan, UT, United States), and handled in a sterile environment [56]. The tissue was washed three times with PBS (phosphate buffered saline), then assembled in the cell culture plate, and cut into small pieces. The small pieces of endometrial tissue were placed in 5 mL of 0.25% trypsin, supplemented with 0.25 mg/mL collagenase Type I (Sigma-Aldrich, St. Louis, MO, USA), and incubated at 37°C on a rotating platform for 1 h. Finally, after washing three times with PBS, 10-mL growth medium (supplemented with 10% fetal bovine serum and 1% penicillin-streptomycin) was added to the pelleted cells and plated into a 10-cm cell culture dish, then cultured at 37°C and 5% CO_2_. Cells were monitored daily by light microscopy, and the culture medium was changed every 2–3 days. Cells are usually visible after 24–48 h, when they reach 75–80% clustering. Trypsin (0.25%) was used to passage the cells.

### Endometrial cancer cell lines culture

Endometrial carcinoma cell lines Ishikawa, HEC-1A, HEC-1B, and KLE were obtained from Shanghai Institute for Biological Sciences, Chinese Academy of Sciences. All cell lines were cultured in complete growth medium, DMEM/F12 (Gibco BRL, Rockville, MD) supplemented with 10% FBS (Gibco BRL, Rockville, MD) and 1% antibiotics, and maintained at 37°C and 5% CO_2_.

### Isolation of KLE and Ishikawa cell subclones

KLE and Ishikawa cells at 75–80% confluency were collected and diluted to a density of 10 cells/mL with medium, then seeded into 96-well plates at 0.1 mL per well. After 1 week of culture at 37°C and 5% CO_2_, single clones from a well were chosen and marked, and two or more clones from any well were excluded. After 3–4 weeks’ culture, we isolated 28 cell subclones from KLE cells, identified as KLE-1 to KLE-28, and 23 subclones were obtained from Ishikawa cells, identified as ISK-1 to ISK-23. The electrophoretic migration rates of these subclones were measured using a cell electrophoresis instrument (DY-100, from College of Life Science, Shandong University, China). The invasion and proliferation abilities of the different invasive subclones were analyzed by *in vitro* and *in vivo* functional cell assays. All data were expressed as mean ± standard error (SE).

### Endometrial cancer tissue samples

Human endometrial tissue samples (*n* = 240) were collected with patients’ informed consent. Endometrial carcinoma specimens (*n* = 200) were obtained from the Department of Pathology, Shandong Provincial Hospital. All patients with endometrial cancer were diagnosed according to the revised International Federation of Gynecology and Obstetrics (FIGO) staging system (stage I, 78 cases; stage II, 65 cases; stage III, 33 cases, and stage IV, 24 cases). Preoperative radiation or chemotherapy was not accepted by all patients with endometrial cancer. Forty normal endometrial tissue samples, obtained by surgical hysterectomy, were acquired from the Department of Pathology, Shandong Provincial Hospital. All patients agreed to a regular follow-up. During the study period, 8 patients were lost, and 20 patients died. The follow-up period was between 2 and 7 years at the end of 2014. The study was approved by the Institutional Medical Ethics Committee of Shandong University.

### Immunohistochemistry (IHC) and Immunocytochemistry (ICC)

For IHC, formalin-fixed, paraffin-embedded endometrial tissues were sliced at a thickness of 5 μm. All sections were dewaxed in xylene and rehydrated in ethanol. After that, antigen retrieval was accomplished in a microwave oven for 15 min with 0.01 M citrate buffer, pH 6.0. For ICC, cells at log phase were seeded into a cell culture plate covered with coverslips. After 24 h, coverslips were gathered and fixed with 95% ethanol for 30 min. Following the protocol for the Streptavidin-Peroxidase Detection Kit (ZSGB-BIO), both sections and coverslips were incubated with 3% hydrogen peroxide (H_2_O_2_) for 30 min to quench endogenous peroxidase activity, and then incubated with rabbit anti-human fibulin-4 antibodies (ab125073, Abcam), diluted 1:200, at 4°C overnight. After washing with PBS, sections and coverslips were incubated with the anti-rabbit biotin-conjugated secondary antibody for 30 min at 37°C, and finally stained with the enzyme substrate 3, 3′-diaminobenzidine tetrahydrochloride (DAB, Sigma-Aldrich, St. Louis, MO, USA). Human ovarian carcinoma paraffin-embedded sections (fibulin-4-positive) were used as positive controls [15]; the negative control was PBS in place of the primary antibody. Brown granules appearing in the cytoplasm or stroma were considered to be immunoreactivity of fibulin-4 [57].

### Immunohistochemistry (IHC) and Immunocytochemistry (ICC) analysis

The percentage of stained cells and the staining intensity were used to assess fibulin-4 expression in IHC and ICC experiments. The percentage of positively stained cells was assigned a score from 0 to 4 (score 0, 0% cells stained; score 1, 1–25% cells stained; score 2, 26–50% cells stained; score 3, 51–75% cells stained; or score 4, 76–100% cells stained). The staining intensity of fibulin-4 was assigned a score from 0 to 3 (score 0, negative; score 1, weak; score 2, moderate; or score 3, strong) [58]. Adding together the intensity and percentage scores gave a total staining score (0–7), and scores of 0, (1–3), (4–5), and (6–7) were translated into the sum indexes (−), (+), (++), and (+++), respectively [58]. For statistical analysis, sum-indexes (−) or (+)were considered low expression of fibulin-4, while (++) or (+++) were considered high expression of fibulin-4. Each tissue section was analyzed by three pathologists independently.

### RNA interference and overexpression transfection

The overexpressed fibulin-4 lentivirus vector and fibulin-4 small hairpin RNA (shRNA) as well as a negative control were obtained from GeneChem Inc (Shanghai, China). According to the manufacturer's instructions, target cells were plated in a 24-well plate and incubated at 37°C in a CO_2_ incubator for 24 h, and then infected by adding viral stock at a multiplicity of infection (MOI) of 100. Cells were incubated at 37°C with 5% CO_2_ overnight. To avoid cell toxicity, the transfection mixture was removed, and new complete medium was added. After further 48 h incubation at 37°C with 5% CO_2_, transfected cells were observed using fluorescence microscopy. Transfection efficiency was detected by western blotting, real-time quantitative RT-PCR, and ICC.

### Quantitative real-time-polymerase chain reaction (RT-qPCR)

Total RNA was extracted using Trizol reagent (TaKaRa Biotechnology), and cDNA was reverse-transcribed from total RNA using a SYBR^®^ Premix Ex Taq^TM^ kit (TaKaRa Biotechnology). Each well (20 μL reaction volume) contained 10 μL Power SYBR Green PCR master mix (TaKaRa Biotechnology), 0.8 μL of each primer (final concentration 0.2 μM), 2 μL template, and 6.4 μL DNAse/RNAse-free water (Sigma-Aldrich). Three wells were used for each template as biological replicates. PCR was performed using the LightCycler^®^480 System (Applied Biosystems Inc.; Thermo Fisher Scientific, Inc.). Specific primers were designed using LightCycler^®^ Probe Design software (Roche Diagnostics, Basel, Switzerland) and synthesized by Takara Biotechnology Co., Ltd. The sequences of primers were as follows: fibulin-4: 5′-GCTGCTACTGTTGCTCTTGGG-3′, 5′-GGGATGGTCAGACACTCGTTG-3′; E-cadherin: 5′-GGATTGCAAATTCCTGCCATTC-3′, 5′-AACGTTGTCCCGGGTGTCA-3′; N-cadherin: 5′-GTAGCTAATCTAACTGTGACCGATAAGG-3′, 5′-TTGGTTTGACCACGGTGACTAA-3′; vimentin: 5′-GCAGGAGGCAGAAGAATGGTA-3′, 5′-GGGACTCATTGGTTCCTTTAAGG-3′; Snail: 5′-TCGGAAGCCTAACTACAGCGA-3′, 5′-AGATGAGCATTGGCAGCGAG-3′; Slug: 5′-TGTGACAAGGAATATGTGAGCC-3′, 5′-TGAGCCCTCAGATTTGACCTG-3′; Twist: 5′-AGCAAGATTCAGACCCTCAAGCT-3′, 5′-CCTGGTAGAGGAAGTCGATGTACCT-3′; β-actin: 5′-CCACGAAACTACCTTCAACTCCA-3′, 5′-GTGATCTCCTTCTGCATCCTGTC-3′.

### Western blotting

Cells were lysed on ice in RIPA (radio-immunoprecipitation assay) buffer containing 1 mM phenylmethylsulfonyl fluoride (PMSF). Samples (40-μg protein per lane) were separated by sodium dodecyl sulfate polyacrylamide gel electrophoresis (SDS-PAGE), transferred to polyvinyl difluoride (PVDF) membranes, and blocked with 5% bovine serum albumin (BSA). Membranes were then incubated with primary antibodies (E-cadherin sc-8426, N-cadherin sc-7939, Vimentin sc-6260, Santa Cruz; fibulin-4 ab125073, Snail ab167609, Slug ab27568, Twist ab50887, β-catenin ab32572, C-myc ab32072, Cyclin D1 ab134175, Notch1 intracellular domain (NICD) ab83232, HES 1 ab71559, HEY L ab154077, Abcam) at working dilutions of 1:1000 at 4°C overnight. On the next day, membranes were incubated with secondary antibody for 1 hour at room temperature, and blots were developed using the enhanced chemiluminescence method (Pierce™ ECL Western Blotting Substrate; Thermo Fisher Scientific, Inc.).

### Growth curves

After trypsin digestion, cells in log phase were collected, seeded into 24-well plates (1 × 10^4^ cells/well) and cultured at 37°C and 5% CO_2_. Cells from 3 wells were counted every day, and the average was obtained for 7 consecutive days. Growth curves were prepared using the average number of cells from each day.

### Soft agar colony formation assay

Cells were harvested and suspended in culture medium. DMEM (1.5 mL) supplemented with 20% FBS was mixed with 1.5 mL 1.2% agar and solidified in 3.5-cm dishes to form the bottom layer. Next, 1.5 mL of 0.7% agar was mixed with 1.5 mL DMEM (20% FBS) and 200 μL cell suspension (containing 600 cells), and this mixture was immediately added to the dishes with solidified bottom layer. The assay was performed in triplicate, and all dishes were incubated for 14 days at 37°C and 5% CO_2_. A cluster of ten cells or more was considered as a colony, detected using an inverted microscope (Nikon Eclipse). The dish was divided into 4 quadrants using horizontal and vertical lines; cells were counted in each quadrant and the center of the dish in a single viewing field, and the average was calculated and expressed as mean ± SE.

### Cell invasion assay and migration assay

The cell invasion assay and migration assay were performed using the Boyden chamber as described by Albini [59]. Boyden chamber assay was based on a chamber of two medium-filled compartments separated by a microporous membrane. In general, cells are placed in the upper compartment and are allowed to migrate through the pores of the membrane into the lower compartment, in which chemotactic agents are present. Matrigel is the trade name for a gelatinous protein mixture secreted by Engelbreth-Holm-Swarm (EHS) mouse sarcoma cells produced and marketed by Corning Life Sciences and BD Biosciences. Matrigel resembles the complex extracellular environment found in many tissues and is used by cell biologists as a substrate (basement membrane matrix) for culturing cells. Polyvinylpyrrolidone-free polycarbonate (PVPF) Boyden chamber membranes were coated with 50 μL of 1:3 Matrigel dilution. The cell suspension (200 μL, 2 × 10^5^ cells) was seeded into the upper chambers. Filtered, serum-free NIH3T3 culture medium (600 μL) was added to the lower chamber as a chemotactic factor, and the Boyden chambers were incubated at 37°C for 24 h. Non-invading cells were cleaned from the upper surface, and cells on the lower surface were fixed with 95% ethanol, stained with hematoxylin and eosin (H&E), and counted in five random high-power fields (HPF) using an inverted microscope. The assay was performed in triplicate. At the same time, a cell migration assay was performed as above, without the Matrigel coating. All data were expressed as mean ± SE.

### Tumor xenografts in nude mice

BALB/C-nu/nu nude mice were purchased from the National Resource Center for Rodent Laboratory Animal of China. For each group, 5 mice were injected subcutaneously, or through the tail veins, with 5.0 × 10^6^ fresh cells. The mice were maintained in a sterile animal facility, fed with sterile pellet feed and autoclaved tap water, and monitored daily for tumor growth. After 2 months, the mice were killed; the tumors were dissected, and lung tissues were processed into paraffin-embedded sections for H&E staining. Using a vernier caliper, tumor volume was calculated according to the formula of V = length × width^2^ × 0.25. The average values were expressed as mean ± SE. This animal experiment was approved by the Institutional Animal Care and Use Committee, and was in compliance with all regulatory guidelines.

### Statistical analysis

IHC data were analyzed by χ^2^ test. A two-tailed *t*-test was performed to compare the means between two groups, and a one-way analysis of variation was used to compare the means among three groups. The data was analyzed using SPSS software version 13.0 (SPSS Inc., Chicago, IL, USA). *P* < 0.05 (two-sided) was considered statistically significant.

## SUPPLEMENTARY MATERIALS FIGURES


